# A Design of the Ecotourism Individualized Route Planning System Based on the Ecological Footprint Model

This article has been retracted.

**DOI:** 10.1155/2022/6342696

**Published:** 2022-06-22

**Authors:** Hengxiu Lv

**Affiliations:** Qingdao Huanghai University, Qingdao, Shandong 266555, China

## Abstract

In this study, aiming at the huge amount of information in the tourism field, the pressure of ecological environment, and tedious personalized route planning, an ecotourism personalized route planning system based on the ecological footprint model is designed. In order to recommend routes that meet the time limit and the starting and ending points of the user's choice, the tourist route recommendation problem is studied as a directional problem on the basis of comprehensively considering the popularity of scenic spots and the user's interest preferences as the scenic spots score. The scenic spot scoring strategy is scenic spot scoring, and the iterative local search strategy is used to plan tourist routes according to the optimization goal with the largest route score, and improve the real tourist routes, food, and accommodation strategies. On the basis of launched tourist routes, they recommend tourists' favorite food and accommodation. The model finally completes the fine arrangement of scenic spots, food, and accommodation in the whole tourist route. The system test results show that the system has obvious advantages in personalized path planning effect, excellent user feedback effect, and certain application value.

## 1. Introduction

With the rapid development of economy and the gradual improvement of people's living standards, holiday tourism has become the choice for most people to reduce stress and liberate themselves [1]. Tourism, as a “smokeless industry” in the early 21st century, has promoted the rapid development of the economy. The scale of the tourism industry is constantly expanding, and the industrial system is becoming more and more perfect. However, with the development of tourism, it also brings many resource and environmental problems. Due to long-term neglect of protection and blind development, great ecological environment pressure has been generated [2]. Therefore, how to realize the sustainable development of tourism under the premise of protecting the ecological environment has become a topic of great concern. Because China's ecotourism planning has not been carried out for a long time, most of ecotourism planning follows traditional tourism planning ideas, and the ecotourism concept is not deeply reflected, and the planning principles and methods need to be further studied and deepened [3]. With the extensive use of information technology, the number of Internet users has increased dramatically, and e-commerce has become a giant in the market, which has promoted the economic development of tourism e-commerce enterprises. Users' choices are also facing diversified choices, and tourism route planning is a very important factor in self-help tourism planning [4]. Various travel recommendation websites and forums on the Internet provide users with rich information and discussion platforms for them to refer to and discuss the itinerary. Faced with a huge amount of information, users usually need to spend a lot of time and energy to obtain and meet their own needs. In the past, the personalized tourism planning system was more convenient to get tourism information, but there were a large number of online tourism websites with large price differences. In order to get routes that meet their own needs, tourists must compare the schemes and prices of several tourism websites before making a choice [5].

With the differentiation of market demand, public participation and the requirements of sustainable development, the concept of ecotourism has been accepted by more and more scenic spots [6]. Tourism is developing rapidly, and the growth rate of tourism in many provinces exceeds that of other industries. Among them, the market demand and enhancement speed of ecotourism are particularly obvious. However, in today's ecotourism market in China, due to the lack of standardized management, the development of ecotourism projects has no rules to follow [7]. At present, with the continuous improvement of Internet technology, the degree of cross-integration between tourism and the Internet has gradually deepened. The tourism industry is developing towards intelligence and information technology. Online tourism services, such as online marketing, online booking, and online payment, are becoming more and more popular, and the online tourism market is maturing [8]. As a new form of tourism, ecotourism has become a hot international tourism project in recent years. However, due to the late introduction of the concept of ecotourism, the construction of ecotourism areas also started late in China [9]. However, in recent years, with the increasing expectations of tourists for ecotourism and the expanding market scale, the upsurge of building ecotourism areas has arisen all over the country, and ecotourism planning projects have sprung up like mushrooms after rain [10]. The main problem of the services provided by existing tourist websites is that most of the products provided by them are provided by travel agencies, and tourists cannot participate in the planning of scenic spots, food, and accommodation in tourist routes. According to the tourists' personal preferences, characteristics, needs, and categories, providing tourists with travel itinerary planning services can better meet the personalized needs of tourists in the current tourism market [11]. On the basis of the ecological footprint theory and the calculation model, this paper designs an ecotourism personalized route planning system.

Tourism is a lifestyle with high demand and consumption of natural resources, so if certain measures are not taken in developed tourism areas, environmental problems will be caused. The development of tourism not only needs the support of environmental carriers but also may affect the healthy development of the environment [12]. The business model of economic development at the expense of destroying the environment is unsustainable, which will seriously exceed the carrying capacity of the environment, cause undue losses to human society, economic development, and cultural activities, and have adverse effects. Therefore, it is of great significance to study the design of the ecotourism personalized route planning system based on the ecological footprint model [13]. At present, there is a lack of detailed division of travel time in travel route recommendation, and less consideration is given to the individual needs of users. The method of ecological footprint analysis is widely used, which involves the research progress of all aspects of tourism. Relevant professors and scholars analyze the sustainable development of ecological environment according to this method, and analyze the development status and bearing capacity of scenic spots through the calculation data of ecological footprint [14]. Based on the study of the ecological footprint model, this paper designs and develops a set of personalized tourism route planning systems. The system can provide users with services, such as tourist route planning, tourist information inquiry, and tourist attractions recommendation. Using photos containing geographic location information and shooting time information, the historical tourist footprints of users are excavated, and according to the historical tourist footprints of each user, the visiting time of users in scenic spots and the popularity of each scenic spot are obtained. Then, the user's interest preference is obtained based on the user's visit time in the scenic spot, and the user's interest preference and popularity of the scenic spot are transformed into the rating of the scenic spot.

## 2. Related Work

Literature [15] holds that the development of the tourism route planning system based on user-generated data will promote the development of text mining, route recognition, image analysis, and statistical machine learning theory. Literature [16] puts forward a real-time planning algorithm for tourist routes. This algorithm uses a dynamic planning algorithm and considers factors, such as stay time, travel season, and user preference, and realizes real-time travel route planning. Through searching and mining user-generated data in the field of tourism, a system is built to help users summarize and analyze previous travel data and experiences, and provide services for users interactively [17]. In order to solve the problem of time wasted in tourist routes, a cuckoo search was used to optimize the time spent on routes [18]. Literature [19] collates and analyzes the current research situation of tourist route recommendation at home and abroad, and puts forward a personalized tourist route recommendation model by using the photo data with spatio-temporal information in view of some shortcomings in the existing research. Then, we recommend tourist routes that meet our individual needs for users. Literature [20] pointed out that in tourism development, the protection of the ecological environment and the development of the local tourism economy should be maintained at the same time, and the adverse effects of human activities in tourism development on tourism destinations should be reduced, and the tolerance of local resource development should also be reduced to a certain extent. Literature [21] pointed out how to measure and analyze the damage of tourism to the ecological environment and control it on the basis of quantitative analysis, and how to develop the sustainable development of the tourism industry which has become the key research object in the field of tourism research in recent years. Literature [22] makes use of travel notes to explore the features of different scenic spots, and combines these features with the interests of users and scenic spots. Based on this tourism information, the tourism-related knowledge is excavated and personalized travel routes for users were planned. In order to help users to plan tourist routes automatically and save time and energy, literature [23] systematically proposed an automatic tourist route planning system based on user-generated data. On this basis, the real-time route guide inside scenic spots is given.

Based on the previous studies, this paper analyzes the main ideas of current tourist route recommendation and summarizes the methods of current tourist route recommendation. At the same time, it also finds the shortcomings and defects in current tourist route recommendation. The existing tourist route recommendation process lacks the consideration of users' personalized needs and the arrangement of users' travel time. Based on the study of the ecological footprint model, a set of personalized tourism route planning system is designed and developed. The system can score all scenic spots uniformly according to the preference information of scenic spots type input by tourists. In order to add the historical tourist data to the scoring model, this part uses the collaborative filtering algorithm based on users to revise the scenic spots score, which can make the scenic spots score more accurate. The tourism route planning software system is realized. The system adopts responsive webpage layout, which can meet the interactive access mode of users' web and mobile applications, and greatly improves the user experience.

## 3. Methodology

### 3.1. Ecological Footprint Model

With the development of social economy and the change of residents' consumption patterns, the natural ecosystem is under increasing pressure, and ecological security becomes particularly important. At present, with the rapid development of tourism, the direct and indirect impacts on the local ecological environment have seriously affected the balance and sustainability of the tourist destination ecosystem. The ecological footprint is also called “ecological occupation” [24]. The ecological footprint model, as a model to measure the degree of sustainable development, has been widely recognized by academic circles in recent years, and scholars have also made relevant research by applying the tourism ecological footprint model. The ecological footprint is a method to quantitatively analyze the damage and utilization degree of natural resources caused by various human activities and the carrying capacity of natural resources in a certain area.

The ecological footprint is mainly used to express tourists' consumption of natural capital by the ecological productive land area, and compared with natural capital that the region can actually provide, to measure the sustainable development of the regional tourism industry [25]. Because everyone wants to consume the products and services provided by nature, which will have an impact on the Earth's ecosystem, it is of great significance to measure the gap between human demand for natural ecological services and those provided by nature. The calculation of the ecological footprint is based on two basic facts. ① Human beings can determine the vast majority of resources they consume and the amount of waste they produce. ② These resources and waste streams can be converted into corresponding biological production areas. Ecological footprint calculation can be expressed by the following formula.

(1) $$\begin{array}{c} EF=N\times e_{f}\\ =N\times \Sigma r_{i}\times A_{i}=\times \Sigma r_{i}\times \left(\frac{c_{i}}{p_{i}}\right), \end{array}$$

where *EF* is the total ecological footprint. *N* is the total population of the region. *e*_*f*_ is the per capita ecological footprint. *i* is the type of the consumption item. *r*_*i*_ is the equilibrium factor of the *i*th consumption item. *A*_*i*_ is the actual ecological productive land area per capita occupied by the consumption item *i*. *c*_*i*_ is the per capita annual consumption of the item *i*. *p*_*i*_ is the global average annual output per unit area of the *i*th consumption item.

The ecological footprint analysis method mainly focuses on analyzing and measuring the consumption of natural capital from the perspective of intuitive biophysical quantities [26]. The degree of sustainable development of energy, which can explain the loss of resources in the ecosystem under the human consumption and transformation, has the advantages of visible model, simple and clear calculation, and strong operability. This makes ecological footprint analysis easy to accept and understand in the field of ecological compensation, and has a wide application range. By analyzing the ecological footprint of tourism from different sides, analyzing the influence of tourists on scenic spots, scientifically planning scenic spot facilities, using energy-saving equipment, promoting the healthy development of protected areas, and reasonably determining the scale and scope of building tourist destination facilities.

To measure the sustainable development of a region's tourism industry, an index with high credibility is urgently needed. This index should not only cover all the services and resources consumed in tourism activities, but also not conflict with other industries. At the same time, the calculation method should be as concise as possible, and the data needed for calculation can be easily obtained. In order to calculate the ecological footprint of tourism, the facilities in tourist attractions will be analyzed in detail, and the near-accurate values will be recorded, and such energy as tourism consumption and services will be converted into a productive land area [27]. The main elements of tourism activities include six categories of ready-to-eat, accommodation, transportation, travel, shopping, and entertainment, so the calculation of the tourism ecological footprint mainly includes six parts: tourism transportation, tourism accommodation, tourism catering, tourism shopping, leisure, and sightseeing. The framework of tourism route planning is shown in Figure 1.

Ecological footprint analysis mainly involves ecological productive land, ecological carrying capacity, and ecological surplus. Eco-productive land can comprehensively compare the equivalent relationships of four different types of land, such as grassland, forest, water area, and built-up land, through the determination of yield factors and equilibrium factors, and transform human production, and consumption activities into six types of land quantitative calculation. Ecological productive land refers to: firstly, it has certain biological productivity, and secondly, it belongs to the surface space in the study area. Because it is always closely related to the surface of the Earth in the productive process of living things, the calculation and analysis of the ecological footprint can be replaced by the surface area of the Earth.

Tourism ecological footprint is the application of the ecological footprint theory in tourism and tourism research, which refers to the area of bioproduction land that can continuously provide various resources related to tourism activities and consume wastes to tourists of a certain scale during tourism activities. In the calculation of the tourists' tourism ecological footprint, the floor area of various project-related facilities and various resource consumption items are finally converted into the land area. The method of expressing the tourism ecological footprint by the productive land area is relatively simple, easy to count and compare among different categories, and convenient to calculate the sum of the total tourism ecological footprint of different projects. Ecological carrying capacity means the bearing degree of scenic spots, that is, the concept of the maximum load. It refers to the sum of e ecological productive land that the region can provide for human beings, and the calculation formula is

(2) $$\begin{array}{c} EC=N\times e_{c}\\ =N\times \Sigma a_{i}\times y_{i}\times r_{i}, \end{array}$$

where *y*_*i*_ is the yield factor. *r*_*i*_ is the equilibrium factor. *a*_*i*_ is the biological productive area per capita. *N* is the population number. *e*_*c*_ is the per capita ecological carrying capacity. EC is the total ecological carrying capacity.

Ecological carrying capacity, the ability of self-regulation and self-maintenance of the ecosystem in a certain region, and the ability of ecological productive land in a certain region to accommodate human production, life, and consumption. With the continuous development of society, energy consumption, and non-renewable resources are gradually decreasing, and human society is facing an unprecedented ecological crisis. Therefore, we should develop new energy sources that are pollution-free and recyclable, so as to make the local area develop orderly and continuously. The ecological evaluation index system of tourist destinations is shown in Figure 2.

According to the relevant data of various land areas in the study area, the ecological carrying capacity of this area can be calculated. Because there are differences in biological productivity and resource endowments in different countries or regions, it is necessary to transform them into adjusted ecological carrying capacity through equilibrium factors and yield factors. Ecological surplus can also judge the rationality of business activities and personal activities. When ecological productive land is less than the ecological carrying capacity, the ecological deficit indicates that ecological productive land cannot carry the human survival, life, and consumption activities. In the long run, there will be serious consequences. Once the ecological deficit is serious, the self-regulation ability of the ecosystem cannot repair the destroyed natural environment, and the imbalance of the ecological environment will inevitably lead to serious consequences, which will have a serious impact on human production, life, and consumption.

### 3.2. Design of the Ecological Personalized Route Planning System

The concept of “ecotourism” originated from green tourism or natural tourism, which originally refers to tourism based on the natural environment. Ecotourism advocates “respect” and “listening” and respects the heterogeneity of nature. The two basic characteristics of ecotourism are: the object of tourism is the natural ecological environment, and the way of tourism does not damage the natural ecological environment. Ecotourism is a kind of diversified and highly selective tourism activity, which has certain selectivity for activities, facilities, and tourists. To go to nature, you do not need a lot of high-grade hardware facilities. Ecotourists should have a higher level of knowledge and comprehensive quality, and at the same time, they can have greater initiative and randomness in tourism activities.

Ecotourism has three core standards. ① Nature is the main attraction, including cultural attractions associated with the natural environment. (2) Focus on the right to learn or appreciate resources themselves, instead of using these resources as a venue for other activities. ③ Sustainability. Ecotourism is often confused with natural tourism. In fact, ecotourism is a special form of natural tourism. Although they have similarities in some aspects, such as the types of destinations, their influence on environmental protection, and local social culture, they are essentially different. There are differences between ecotourism and general mass sightseeing in many aspects, such as tourist destinations, facility level requirements, ownership of facilities, and so on.

Landscape ecology is a science that studies the structure, function, and dynamics of landscape. For the spatial pattern and its changes in landscape structure, landscape ecology has worked out a series of qualitative and quantitative indicators. These characteristics have a great influence on the distribution, movement, and persistence of biological species. Ecotourism planning is a branch of tourism planning, which is of great significance to the development and construction of ecotourism. Tourism route planning is a research subject with strong subjectivity. The goal is to provide users with more satisfactory personalized tourism routes, directions, and road guides during the journey. Tourism route planning is a very important link for users to prepare for tourism. The route search often adopts different strategies because of different targets and search terms. Getting high-quality tourism information efficiently from massive Internet data, deeply analyzing users' consumption habits and their own needs, and setting tourism strategies are the core fields of Internet technology research at present.

We use $\bar{V}\left(a\right)$ to denote the average visit time of any user at the scenic spot a, then the average visit time required for each scenic spot a is shown in the following formula:

(3) $$\begin{array}{c} \bar{V}\left(a\right)=\frac{1}{n}\sum_{u\in U}\sum_{a_{x}\in S_{u}}\left(t_{a_{x}}^{l}-t_{a_{x}}^{r}\right)\sigma \left(a_{x}=a\right),\;\forall a\in A. \end{array}$$

Among them, *U* represents the set of all users, and the number of users who have visited the scenic spot a in the user set *U* is denoted as *n*, $\sigma \left(a_{x}=a\right)=\left\{\begin{array}{cc} 1, & a_{x}=a,\\ 0, & \text{other}. \end{array}\right.$

The user's interest preference is the user's liking for a certain type of the scenic spot, so formula (4) is used to calculate the user u's liking degree for the scenic spot with the category attribute *c*.

(4) $$\begin{array}{c} \text{Int}\left(u,c\right)=\sum_{a_{x}\in S_{u}}\frac{\left(t_{a_{x}}^{l}-t_{a_{x}}^{r}\right)}{\bar{V}\left(a_{x}\right)}\sigma \left({\text{Cat}}_{a_{x}}=c\right),\;\forall c\in C, \end{array}$$

where Cat_*a*_ represents the category attribute of attraction *a*, $\sigma \left({\text{Cat}}_{a_{x}}=c\right)=\left\{\begin{array}{cc} 1, & {\text{Cat}}_{a_{x}}=c,\\ 0, & \text{other}. \end{array}\right.$

The construction of the index system in this paper follows the following four principles. ① Scientific nature. ② Operability. ③ Clarity. ④ Combination of qualitative and quantitative. The selected index reflects the natural landscape resources and the ecological environment of tourist destination as much as possible, and can reflect whether the tourism products of scenic spots have reached the characteristics of ecotourism products. A background management system is a management platform for system administrators to maintain information; the web server mainly provides data services for users, and users only exchange data with the web server. The real-time data of weather, scenic spots, and other information is obtained through the web server in the related information network server and the internal server of the meteorological service network through the interface system and fed back to users. To distinguish it from routes between scenic spots, the routes inside scenic spots are called routes. The so-called path is connected by photos containing geographic information. The original tourist footprints uploaded by users are usually incomplete, so they are called incomplete paths in this paper.

In order to improve the speed of the algorithm, it must be able to quickly evaluate whether the scenic spot can be inserted into the tourist route. It takes a long time to check whether other scenic spots can be inserted, but we can record the wait and maxShift of scenic spots already in the tourist route by the recording value to reduce computation time. wait is the waiting time and *a*_*i*_ is the time when tourists arrive at the scenic spot *i*. When the tourist arrives before the opening time of the scenic spot, wait_i_ is *O*_*i*_ minus *a*_*i*_. If the arrival time is within the opening time window of the scenic spot, the value of wait_i_ is 0, as shown in the following formula:

(5) $$\begin{array}{c} {\text{wait}}_{i}=\max\left[0,O_{i}-a_{i}\right]. \end{array}$$

maxShift is the maximum delay time for completing the current service under the condition that the time window constraints of current line attractions are met. The value of maxShift_*i*_ is equal to the sum of the waiting time for next attraction and the maximum delay time until the closing time of last attraction, as shown in the following formula:

(6) $$\begin{array}{c} {\text{maxShift}}_{i}=\min\left[C_{i}-s_{i},{\text{wait}}_{i+1}+\max\;{\text{Shift}}_{i+1}\right]. \end{array}$$

The definition of maxShift reduces the computational complexity of insertable sights to linear, making the algorithm faster. shift_*j*_ represents the time shift after inserting the scenic spot *j* between scenic spots *i* and *k*, as shown in the following equation:

(7) $$\begin{array}{c} {\text{shift}}_{j}=t_{ij}+{\text{wait}}_{j}+T_{j}+t_{jk}-t_{ik}. \end{array}$$

The scenic spot module of the system can retrieve the overall information of scenic spots, including the situation of scenic spots and information near scenic spots. This module provides users with scenic spot inquiry, and users can enter tourist destinations in this module. The challenge of naming scenic spots with place names table lies in how to distinguish common place names from scenic spots names. The same latitude and longitude may correspond to several place names, some are scenic spots and some are ordinary place names. How to automatically screen out the scenic spots is a great challenge. To solve this problem, we count the number of times each place name appears in travel notes. The more times, the greater the probability that the place name is a scenic spot. In this way, we will count the correlation coefficient between each place name and the scenic spot, and then use this coefficient and the place name table to name the scenic spot.

Firstly, the algorithm selects a travel route that can be planned, and then selects one of the routes for weather forecast data analysis, evaluate the overall road priority, and finally output the tourism personalized route planning results. The method of evaluating road priority is

(8) $$\begin{array}{c} R=\frac{TP_{X}}{b_{\max}}. \end{array}$$

In the formula, *R* is the driving time under the maximum safe speed *b*_max_ of a certain road section and TP_X_ is an adjustable constant. After sorting and comparing the *b*_max_ of each route, you can get the best and personalized ecotourism itinerary.

In order to generate personalized tourist routes, we need to associate the user's preferences with the characteristics of each scenic spot. The so-called user preference includes two aspects. ① Travel season and ② Individual's preference for tourism. Therefore, in order to connect user preferences with scenic spots, it is necessary to explore the characteristics of related scenic spots. Geographical information, such as the distance between the departure place and the destination, the road grade, and whether there is a toll station on the way, are the core parameters of route planning. Bad weather, such as smog, sandstorm, snow, ice, and so on, should be evaluated and analyzed, and used as a route for users to avoid danger.

The purpose of landmark identification is to identify geographical location that users are interested in. Using pictures containing geographical location information and text information about tourism on the Internet, a list of world-famous scenic spots is mined, and candidate pictures of each scenic spot are obtained from the Internet based on this list. After efficient image matching and unsupervised clustering of candidate images, the landmark visual model is constructed. Finally, the images of each scenic spot are filtered to generate the landmark list and the corresponding visual model.

## 4. Result Analysis and Discussion

Usually, people always take photos in a tourist attraction during their travel, and users also share their favorite photos to social media websites to record their travel history. The quality of the path indicates how close the path inside a scenic spot is to the ideal path. An ideal path can be imagined as a user who keeps taking photos from the moment he enters a certain scenic spot until he leaves, and uploads all the photos he has taken to an online photo album. In other words, an ideal path has a very high photo density and path span. Ecotourism product evaluation is mainly a process of judging whether the tourism products developed in scenic spots meet the ecological standards from the nature of ecotourism products. The products referred to in this paper include sightseeing items, tourism facilities, and tourism services, and evaluation includes the evaluation of ecotourism project development, environmental education system, and facilities construction in mountain-type tourist destinations.

One of the most important factors in personalized travel route recommendation is to consider the user's preference for a scenic spot. The user's preference for a scenic spot is usually influenced by two factors, one is the popularity of the scenic spot, and the other is the user's preference for the type of the scenic spot. We have conducted a wealth of user surveys to evaluate the algorithm of tourism route planning proposed in this paper. The user inputs the travel location, time, travel season, and personal preference for scenic spots, and obtains the recommended route through these inputs. For the generated routes, they will score according to the scoring standard. And according to the individual's wishes, you can arbitrarily change the input, add, or delete scenic spots to obtain personalized travel route recommendations. Users participating in the user survey are only allowed to score the route planning in cities they have been to. In the questionnaire, the tourists' origin and transportation, as well as their diet structure and consumption will be involved. According to the questionnaire, the average travel distance and average travel days of tourists will be calculated.

The standard data is the output standard factor, equilibrium factor, standard value of land productivity, standard data of heat generation, and heat generation of each energy source corresponding to each related value. In order to evaluate the route planning algorithm proposed in this paper, we propose two other comparison algorithms, one is the route planning algorithm using the time estimation method of an incomplete path average, which calculates the typical stay time in scenic spots by calculating the time average of incomplete paths, and the other is the random route planning method, that is, randomly generating scenic spots to visit every day and randomly planning routes. The survey results are shown in the figure. To what extent do the scenic spots in the route express the style and culture of the city, and its representativeness is shown in Figure 3. Diversity is shown in Figure 4. Rationality is shown in Figure 5.

It can be seen from the figure that the route recommended by this method contains more representative scenic spots, and the route is diversified, which reasonably connects representative scenic spots into route planning. Comparatively speaking, although the time estimation method of the incomplete path average can also select representative scenic spots, the very poor estimation result of stay time makes it impossible to recommend a satisfactory route. A stochastic route planning method is the worst route planning method, which can neither pick out representative scenic spots nor organize scenic spots into tourist routes.

Usually, the more users like a scenic spot, the more photos they will take in the scenic spot and the longer they will stay in the scenic spot. Therefore, we get the user's interest preference based on time according to the user's stay time in a specific type of scenic spots, and then, according to the user's time limit and the selected starting point and ending point of play, we build a personalized tourist route recommendation model based on the popularity of scenic spots and the user's interest preference, so as to recommend the tourist route that meets the user's own needs. The experimental results show that the route recommended by considering the popularity of scenic spots and users' interest preferences comprehensively has a higher accuracy and recall rate than only considering the popularity of scenic spots or users' interest preferences. In the composition stage, we need to consider the score of each vertex, the time spent, the score of each edge, and the time spent walking through each edge. In the stage of dynamic route planning, we need to consider how to arrange the N routes with highest scores from these vertices and recommend them to users. It should be pointed out that in route planning, each scenic spot can only appear once in a certain route at most.

Tourists input their preferences for tourist attractions, and then the algorithm engine module according to the planning system calculates and returns the planned tourist routes. The front end receives the tourist route results and displays them through the map. Because each path is composed of several incomplete paths, for any two incomplete paths, to fuse them into one path, we must first find a pair of reference points and think that they were taken at the same time. Therefore, the shooting time of photos in the two paths is moved to the same reference frame, and photos in paths can be merged into a new path in a chronological order. In this way, we can calculate the time cost of a route merged by several incomplete routes, that is, a sample of the stay time inside the scenic spot. The usability of this system is tested by user evaluation. The user evaluates the overall satisfaction of the recommended route, and the result is shown in Figure 6.

From evaluation results, it can be seen that users have the highest overall satisfaction with the recommended route in this paper, which further verifies the practicability of this method. The analytic hierarchy process (AHP) is used for evaluation, which is a systematic and a hierarchical analysis method combining qualitative and quantitative analysis. It is used to solve the weights of multiple targets that obey the overall goal or to solve the weights of multiple factors to the associated multiple target factors. When multiple goals and factors form a step-by-step structure, the analytic hierarchy process can analyze the weight of any level of goals or factors to the previous level of goals or factors, and finally get the weight of the overall goal.

According to the user's preference for information about scenic spots, food, accommodation, and so on, and considering the time distance between scenic spots, the opening hours and closing hours of scenic spots plan several tourist routes for tourists. The typical stay time inside a scenic spot can be estimated by the excavated route inside the scenic spot. In order to evaluate the dwell time estimation algorithm, we choose two comparison algorithms, one is time estimation based on the incomplete path, the other is time estimation based on the Gaussian model. Among them, time estimation based on incomplete paths refers to counting the starting and ending times of incomplete paths provided by all users in a scenic spot, so as to calculate the average time as the typical play time in the scenic spot.

The travel system based on the Android system and the Baidu map, the travel system based on WebGIS technology and this system are used for route planning, and the personalized travel route planning effects of the three systems are tested. Taking the driving safety rate and time consumption of personalized travel routes as the indicators of the route planning effects, the planning effects of the three systems are shown in Figures 7 and 8.

It can be seen from Figure 7 that the route driving safety rate planned by this system is higher, and the route driving safety rate planned based on the Android system and the WebGIS system is lower than this system. The route planned by this system has fewer traffic accidents, lower traffic congestion, and the best planning effect. As can be seen from Figure 8, there are differences in the time-consuming of tourist routes planned by the three systems. In this street, tourist routes planned by the system in this paper can reach the destination with less consumption, while tourist routes based on the Android system and the WebGIS system have higher time-consuming, which shows that tourist routes planned by the system in this paper are the shortest.

The scenic spot scoring strategy transforms the user's preference for scenic spots into the user's rating for scenic spots. The iterative local search strategy plans a route with the highest total score of scenic spots in the travel itinerary for the user, while the search optimization strategy optimizes the travel itinerary time of the iterative local search, so that the time spent on the travel itinerary can be reduced as much as possible. In this chapter, experiments are carried out to compare the optimization effects of different selection strategies on the total route score, and route planning is compared with this system by using the tourism system based on the Android system and the Baidu map, and the tourism system based on WebGIS technology. The results show that the method proposed in this paper can get higher route scores when adopting the elite selection strategy, and has more efficient performance in operation efficiency.

## 5. Conclusion

The rapid development of tourism has undoubtedly produced great economic and social benefits, but at the same time, it has also brought some negative ecological and environmental problems. Tourism is no longer the once called “smokeless industry”. At present, the per capita tourism ecological footprint of many tourist areas has exceeded the per capita ecological carrying capacity, resulting in the ecological deficit and ecological deterioration. The main reason is that the ecological occupation of tourism is growing too fast, that is, the rapid increase of the tourist scale, the expansion of infrastructure, the deterioration of consumption patterns, and so on. In the calculation of six kinds of the tourism ecological footprint, the transportation part basically accounts for a large proportion, and energy consumption included in the transportation calculation part will correspondingly account for a relatively large proportion. Therefore, in order to reduce the consumption of the ecological footprint in scenic spots, we can increase the management from the traffic part, coordinate with other parts, rationally plan and construct traffic land, and reduce the energy consumption per driving distance of sightseeing buses in scenic spots. Eco-personalized route planning and design is the key content in the current study of tourist routes, and it has become a difficult point in the current study of tourist route optimization because of the characteristics of large amount of information and less quantitative data of tourism-related elements. Based on the study of the ecological footprint model, this paper constructs an ecotourism personalized route planning system. The model combines various attributes of tourist attractions, and comprehensively considers three factors of space, time, and tourists' demand in the tourist links, and provides services, such as tourist route design and schedule arrangement for tourists. The experimental results show that the selection strategy proposed in this paper can recommend tourist routes with higher satisfaction for users. However, many practical factors need to be considered in real-life tourism route planning activities, so there is still a lot of work to be performed in the future.

## Figures and Tables

**Figure 1:** Tourism route planning framework.

**Figure 2:** Ecological evaluation index system of tourist destination.

**Figure 3:** Representative evaluation.

**Figure 4:** Diversity evaluation.

**Figure 5:** Rationality evaluation.

**Figure 6:** Comparison of users' overall satisfaction evaluation on recommended routes.

**Figure 7:** Comparison result of driving safety rate.

**Figure 8:** Comparison results of travel route time consumption.

## Data Availability

Data are available upon request.
